# Xingnao Jieyu Decoction Reduces Neuroinflammation through the NF-*κ*B Pathway to Improve Poststroke Depression

**DOI:** 10.1155/2021/8629714

**Published:** 2021-10-23

**Authors:** Dou Wang, Tao Li, Xuefei Han, Weiwei He, Yongmei Yan

**Affiliations:** ^1^Encephalopathy Hospital, Affiliated Hospital of Shaanxi University of Chinese Medicine, West Weiyang Road, Xianyang, Shaanxi 712000, China; ^2^First Clinical Medical College, Shaanxi University of Chinese Medicine, West Weiyang Road, Xianyang, Shaanxi 712000, China

## Abstract

The neuroinflammatory pathway regulated by nuclear factor kappa-B (NF-*κ*B) plays an important role in the occurrence, development, and prognosis of poststroke depression (PSD). The regulatory effect of the traditional Chinese medicine compound Xingnao Jieyu decoction (XNJY) on the NF-*κ*B pathway of PSD is still unclear. This study aimed to observe the effect of XNJY on PSD and explore the molecular mechanism of its intervention in the NF-*κ*B pathway. Middle cerebral artery occlusion (MCAO) and chronic unpredictable mild stress were used to establish a PSD rat model. Body mass measurement, behavioral testing, Nissl staining, ELISA, and Western blot were also performed. XNJY and fluoxetine hydrochloride (Flu) treatment of PSD model rats showed significant antidepressant effects. XNJY and Flu treatment could reduce cortical and hippocampal neuronal damage. XNJY reduced inflammation and restored the levels of IL-4, IL-10, and BDNF. In addition, XNJY showed a significant regulatory effect on the NF-*κ*B pathway and the expression of synapse-related proteins PSD-95 and SYN. These results showed that XNJY could significantly reduce the depressive symptoms of PSD rats, and this reduction may be related to the regulation of the NF-*κ*B signaling pathway to improve neuroinflammation and synaptic function.

## 1. Introduction

Poststroke depression (PSD) is a very common neuropsychiatric disorder after stroke, characterized by depression, loss of interest, anxiety and sleep disorders, and even suicidal thoughts [1, 2]. In a multicenter case-control study conducted in Ghana and Nigeria, the prevalence of PSD was 25.9% [3]. In another Iranian systematic review and meta-analysis study, the prevalence of PSD was 46.9% [4]. PSD has a negative effect on the functional outcome, rehabilitation response, and quality of life of survivors [5, 6]. It is one of the important reasons for the high recurrence, mortality, and disability rates of stroke [7–10]. The pathogenesis of PSD involves the lack of monoamine transmitters in the brain, hypothalamic-pituitary-adrenal axis dysfunction, insufficient neurotrophic factor content, intestinal flora disorders, neuroinflammation, and synaptic plasticity damage [10, 11]. Among them, neuroinflammation and synaptic plasticity damage have a continuous role in the pathogenesis of PSD, and they are believed to be closely related to the occurrence of PSD and other complications.

At present, the treatment of PSD is mainly based on the tricyclic and tetracyclic drugs used in the monoamine hypothesis of depression, as well as norepinephrine and serotonin reuptake inhibitors [12, 13]. Among them, selective serotonin reuptake inhibitors and tricyclic antidepressants are the two most widely studied drugs, and their antidepressant effects were found to be related to the improvement of synaptic plasticity [14]. In addition, patients with depression are often accompanied by elevated inflammatory factors. Some anti-inflammatory drugs could effectively relieve stroke and improve depression symptoms. Certain antidepressants could reduce the level of inflammation in patients with depression. Therefore, reducing neuroinflammation and improving synaptic plasticity are considered potential targets for PSD therapeutic intervention. Nuclear factor-*κ*B (NF-*κ*B) is a classic mechanism that regulates neuroinflammation. The NF-*κ*B pathway caused by inflammation, stress, ischemia, and hypoxia activates and damages synaptic plasticity and affects neurogenesis in the brain [15, 16]. Acute stress-induced NF-*κ*B activation in rat neural stem cells inhibited hippocampal neurogenesis [17]. Similarly, maternal infections affected fetal brain neurodevelopment through the release of NF-*κ*B-regulated proinflammatory activators [18, 19]. Chinese medicine is one of the commonly used complementary and alternative medicine treatment methods for PSD. Under the condition of accurate syndrome differentiation, traditional Chinese medicine has the characteristics of simultaneous treatment of symptoms and root causes, multiple targets, and lighter side effects than Western medicines. XNJY (Chinese herbal medicine compound) is an empirical prescription for the treatment of PSD clinically, with significant clinical effects. In early animal experiments, PSD model rats improved through the BDNF/ERK/CREB pathway and showed a reduction in proinflammatory cytokines after XNJY treatment [20]. In the present study, middle cerebral artery occlusion (MCAO) and chronic unpredictable mild stress (CUMS) were used to establish a PSD rat model to further clarify the molecular mechanism of XNJY in alleviating neuroinflammation and improving PSD.

## 2. Materials and Methods

### 2.1. Reagents and Drugs

XNJY consists of 12 g *Acorus tatarinowii*, 12 g *Polygala*, 30 g *Salvia*, 12 g *Bupleurum*, 15 g *Albizia Julibrissin*, 10 g turmeric, and 10 g *Morinda officinalis*. All Chinese herbal medicines were provided by the Chinese Pharmacy of the Affiliated Hospital of the Shaanxi University of Traditional Chinese Medicine in accordance with the standards included in the Chinese National Pharmacopoeia. The decoction was prepared by placing the mixture in distilled water twice and boiling it at 100°C for 30 min. The obtained herbal juice was concentrated into XNJY-10.5 g/kg treatment group and XNJY-21 g/kg treatment group. Each rat was given 3 mL of gavage soup. Fluoxetine hydrochloride (Flu, #7723A) was purchased from Lilly and Company (Suzhou, China). Nissl Staining Kit (#G1432) is available from Solarbao (Beijing, China). Brain-derived trophic factor (BDNF, #371677828), tumor necrosis factor-*α* (TNF-*α*, #2401582814), interleukin-1*β* (IL-1*β*, #1151662828), interleukin 6 (IL-6, #1331659828), interleukin-4 (IL-4, #1281670828), and interleukin-10 (IL-10, #1381612828) ELISA kits were obtained from Boster Biological Technology Co., Ltd (Wuhan, China). Anti-NF-*κ*B (#BM3932), anti-NF-*κ*B inhibitory protein *α* (I*κ*B-*α*, #bs-0465R), and *β*-actin (#BM0627) were purchased from Boster Biological Technology Co., Ltd. (Wuhan, China) for Western blot. Anti-p-NF-*κ*B (#AF2006) and anti-p-I*κ*B-*α* (#AF2002) were purchased from Affinity Biosciences, Ltd (Changzhou, China). Anti-SYN (#ab32127) and anti-PSD-95 (#ab18258) were purchased from Abcam Limited (Cambridge, USA). Enzyme-labeled goat anti-rabbit IgG (#BA1054) and enzyme-labeled goat anti-mouse IgG (#BA1050) were purchased from Boster Biological Technology Co., Ltd (Wuhan, China).

### 2.2. Animals and Management Procedures

#### 2.2.1. Animals, Grouping, and Intervention

Male Sprague Dawley rats (200 ± 20 g, 7–8 weeks) were provided by the Experimental Animal Center of the Xi'an Jiaotong University School of Medicine. The program was approved by the Animal Protection and Use Committee of the Shaanxi University of Chinese Medicine (Approval No. SUCM20190311001). The rats adapted to feeding for 1 week under standard laboratory conditions (temperature of 22°C ± 2°C, humidity of 55% ± 5%, and 12 h of light/12 h of dark cycle). After MCAO and sham operation were performed, the rats were randomly divided into sham operation, PSD, Flu, and XNJY (XNJY-10.5 g/kg and XNJY-21 g/kg) groups. The sham operation group and MCAO group were given saline intragastrically for 21 days. The PSD group was treated with CUMS and provided with saline intragastrically for 21 days. The Flu group was treated with CUMS and given Flu (2.08 mg/kg) by gavage for 21 days. The XNJY group was treated with CUMS and given different doses of XNJY (XNJY-10.5 g/kg and XNJY-21 g/kg) for 21 consecutive days.

#### 2.2.2. MCAO Model

The MCAO model is a nylon monofilament thread (#2541, Henan, China) coated with silica gel through the right internal carotid artery to the right middle cerebral artery [21]. It was occluded for 60 minutes and then taken out after the MCAO operation. All rats had free access to food and water for 2 days in a stress-free cage. The Zea-Longa 5-point method was used to evaluate the neurological deficit score of the MCAO model rats, and the surviving rats with scores of 1–3 were selected for follow-up experiments.

#### 2.2.3. CUMS Model

The CUMS model was prepared using Willner's method [22, 23]. The rats were exposed to one stressor per day to induce depression for 21 consecutive days. These stressors had seven kinds; each stimulus was repeated three times irregularly during the treatment period, and the stressors were different for the next 2 days. All stressors included food and water deprivation (24 h), wet cage (200 mL of water per 100 g litter, 24 h), tail pinching (1 min), forced swimming (4°C, 5 min), electric shock ((0.9 mA, 15 s) × four times), day and night upside-down (24 h), and shaking the cage (200 Hz, 5 min).

### 2.3. Rat Body Weight and Depression-Like Behavior Assessments

#### 2.3.1. Body Weight Assessment and Sucrose Preference Test

Body weight and sugar water consumption were measured on days 1 and 21 of the experiment. The reward behavior of rats was evaluated using the sucrose preference test. The animals were deprived of food and water for 24 h. Experiments were conducted by giving one bottle of drinking water and one bottle of 1% sucrose water (weighed in advance). After 1 h, the bottle was taken out and weighed. The following formula was used to calculate the result: sucrose intake/(sucrose intake + water intake).

#### 2.3.2. Forced Swimming Test

After the last treatment, a forced swimming test was used to evaluate the desperate state of the rats. The rats were forced to swim alone for 5 min in a glass cylinder (height of 15 cm and diameter of 10 cm) filled with water (25°C ± 2°C). During the test, two blind testers recorded the immobility time of the rats.

#### 2.3.3. Open Experiment

An open box with a black inner wall (bottom of 100 cm × 100 cm and height of 50 cm) was used to evaluate the desperate behavior of rats. The bottom of the box was divided evenly into 25 small squares of the same size. The rat was placed in the center of the box. After the 5-min test, the number of squares crossed by the four paws of the rat was the horizontal score, and the number of standing hind limbs was the vertical score [13]^.^ After the test of each rat was finished, the bottom surface of the square box was cleaned to prevent the remaining information of the animal from the previous test (such as the animal's urine and feces) from affecting the next test result.

### 2.4. Nissl Staining

Nissl staining was used to observe the damage in the cortex and hippocampal neurons. The rats were anesthetized with 10% chloral hydrate, and samples were taken, fixed with 4% paraformaldehyde for 24 h, dehydrated with different concentrations of ethanol gradient, embedded in paraffin, and sectioned. After deparaffinization, toluidine blue was stained, and then the slides were mounted for microscopic examination using a microscope (DP73, Olympus). Images were collected and analyzed. Quantitation of Nissl-stained neurons in each slice of the cortex and hippocampus was blindly observed with five fields of view.

### 2.5. ELISA Determination

An ELISA kit was used to detect cytokines, such as BDNF, TNF-*α*, IL-*β*, IL-6, IL-4, and IL-10, in the rat cortex and hippocampus. Specific steps were carried out in accordance with the instructions.

### 2.6. Western Blot Detection

Western blot was conducted to detect p-NF-*κ*B/NF-*κ*B, p-I*κ*B-*α*/I*κ*B-*α*, PSD-95, and SYN in the rat cortex and hippocampus. The rats were anesthetized, the heart was perfused, and the brain was decapitated. The rat cerebral cortex and hippocampus tissues were separated on ice. Lysate, protease inhibitor, and phosphatase inhibitor were added to the tissues for continuous lysis for 30 min and then homogenized by ultrasound. The lysate was centrifuged at 12000 rpm for 10 min to obtain the supernatant and the tissue protein. The BCA method was used to detect the protein concentration. Then, the sample was added to 5× loading buffer and boiled. The target protein was separated by 10% SDS-PAGE gel electrophoresis, transferred to a PDVF membrane, and blocked with 5% skimmed milk for 1 h. Subsequently, it was incubated overnight with the primary antibody diluted in a certain proportion and then placed on a shaker at 4°C. The PVDF membrane was incubated with the corresponding secondary antibody for 1 h, and the ultrasensitive ECL reagent and gel imaging system were used to emit light and take pictures. ImageJ software, version 2.0, was used to statistically analyze the gray value of protein bands.

### 2.7. Statistical Analysis

Data were analyzed using SPSS software, version 19.0, and expressed as mean ± SEM. Statistical significance was determined using one-way or two-way difference analysis, and multiple comparison analysis was performed using Tukey's test afterward. *P* < 0.05 was considered statistically significant.

## 3. Result

### 3.1. XNJY Increases the Body Mass of PSD Model Rats and Improves Depression-Like Symptoms

The timetable of the experimental procedure is shown in Figure 1(a).  Figure 1(b) shows the body weights of rats in each group on day 22 of the experiment. The weight of the PSD group was significantly reduced (*P* < 0.01) compared with that of the sham operation group. The weight of rats after treatment with Flu and XNJY significantly increased compared with that of PSD model rats (*P* < 0.01).

The sucrose preference test (Figure 1(c)), forced swimming test (Figure 1(d)), and open-air test (Figures 1(e) and 1(f)) were used to evaluate the depression-like symptoms of rats on day 22 of the experiment. Compared with the sham operation group, the PSD group showed significantly reduced sucrose consumption, horizontal movement, and vertical movement, and the immobility time during forced swimming was significantly prolonged (*P* < 0.01). On the contrary, the sucrose intake and spontaneous movement (including horizontal movement and vertical movement) of rats increased significantly after Flu and XNJY treatment, and the resting time during forced swimming was shortened (*P* < 0.01).

### 3.2. XNJY Protects PSD Model Rats from Neuronal Damage

The effect of XNJY on nerve damage was evaluated in the cortex and hippocampus of the PSD group via Nissl staining (Figure 2). A significant loss of Nissl-stained neurons was found in the cortex and hippocampus of the PSD group (*P* < 0.01). Different doses of XNJY and Flu treatment increased the quantitation of Nissl-stained neurons in the cortex and hippocampus compared with those in the PSD group (*P* < 0.05).

### 3.3. XNJY Reduces Inflammation in PSD Model Rats and Restores the Levels of IL-4, IL-10, and BDNF

The levels of IL-6, TNF-*α*, and IL-1*β* in the cortex and hippocampus were measured (Figures 3(a)–3(c)). They were significantly increased in the cortex and hippocampus of the PSD group (*P* < 0.01). Different doses of XNJY reversed these abnormal indicators (*P* < 0.05). Flu treatment downregulated these proinflammatory factors in the hippocampus (*P* < 0.05). However, compared with the XNJY group, the Flu group did not show any abnormal indicators in the cortex.

The levels of IL-4, IL-10, and BDNF in the cortex and hippocampus were also measured (Figures 3(d)–3(f)). Compared with the sham operation group, the PSD group had significantly reduced levels of IL-4, IL-10, and BDNF in the cortex and hippocampus (*P* < 0.01). After different doses of XNJY treatment were administered, these levels in the cortex and hippocampus were significantly restored (*P* < 0.01). Meanwhile, the BDNF level of the cortex and hippocampus increased significantly in the Flu group (*P* < 0.01). Flu treatment modulated IL-4 and IL-10 in the hippocampus, but this effect was not detected in the cortex.

### 3.4. XNJY Regulates the NF-*κ*B/I*κ*B-*α* Pathway in PSD Model Rats

Western blot was used to determine NF-*κ*B, p-NF-*κ*B, I*κ*B-*α*, and p-I*κ*B-*α* in the cortex (Figures 4(a) and 4(c)) and hippocampus to explore the new potential mechanism of the XNJY antidepressant (Figures 4(b) and 4(d)). Compared with the sham operation group, the PSD group exhibited an increase in the p-NF-*κ*B/NF-*κ*B and p-I*κ*B-*α*/I*κ*B-*α* protein ratios (*P* < 0.01). Different doses of XNJY treatment could reduce the levels of p-NF-*κ*B/NF-*κ*B and p-I*κ*B-*α*/I*κ*B-*α* protein ratios in the cortex and hippocampus (*P* < 0.01). Flu treatment downregulated these ratios in the hippocampus (*P* < 0.01) but had no effect in the cortex.

### 3.5. XNJY Regulates Synapse-Related Proteins in PSD Model Rats

Western blot was further used to detect the protein levels of PSD-95 and SYN in the cortex (Figures 5(a) and 5(c)) and hippocampus (Figures 5(b) and 5(d)). The PSD group had lower protein levels of PSD-95 and SYN in the cortex and hippocampus than the sham operation group (*P* < 0.01). Flu and different doses of XNJY treatment could increase these protein levels in both regions (*P* < 0.05).

## 4. Discussion

The antidepressant effect and mechanism of XNJY in PSD model rats were explored. The results showed that XNJY improved depression-like symptoms and reduced cortical and hippocampal neuronal damage. Further research found that XNJY inhibited the NF-*κ*B/I*κ*B-*α* pathway in the cortex and hippocampus, downregulated the levels of IL-6, TNF-*α*, and IL-1*β*, and restored the levels of IL-4, IL-10, and BDNF to reduce inflammation. XNJY also restored the levels of synaptic plasticity-related proteins, such as PSD-95 and SYN, in the cortex and hippocampus of PSD rats. These results indicated that reducing inflammation and improving synaptic plasticity may be importantly related to the antidepressant effect of XNJY.

PSD is the main cause of poor recovery, decreased quality of life, and poor rehabilitation effect in patients [6]. At present, drug therapy is still the main treatment for PSD, despite the drug withdrawal and toxic side effects [24–26]. XNJY soup is a Chinese herbal compound with a great potential in the treatment of PSD. Research showed that XNJY could treat depression by improving rat body weight, sucrose preference, voluntary activity, and resting time during forced swimming. The quality of life of patients with PSD is significantly lower than that of patients with simple stroke, especially in the fields of cognition, emotion, limb function, and social function [27, 28]. PSD and poor neural prognosis may be directly related to neuronal damage or apoptosis after stroke. Reducing neuronal damage, protecting neuronal survival, and promoting neuronal repair and regeneration may be important targets for the prevention and treatment of related diseases after stroke. The Nissl body is a characteristic structure of the neuron cell body. When neurons are damaged, the Nissl body dissolves and disappears [29]. The present study found that the neuron Nissl bodies in the cortex and hippocampus of PSD rats were significantly missing, and XNJY and Flu treatment could increase the number of Nissl bodies in both regions.

The neuroinflammatory response involves the whole process of the occurrence and development of stroke, and it has an adverse effect on complications, including depression [30, 31]. Adjusting the inflammatory response could improve the symptoms of depression after stroke [32]. NF-*κ*B is a transcription factor that accumulates in the cytoplasm in the form of a dimer in a resting state. After activation, it enters the nucleus to regulate gene transcription. I*κ*B-*α* phosphate is activated and degraded to separate NF-*κ*B from it. Phosphate-activated NF-*κ*B enters the nucleus, promotes the increase in IL-1*β* and TNF-*α* levels, and triggers an inflammatory response. Clinical studies have reported that the severity of depression in patients with PSD is positively correlated with the levels of IL-6, TNF-*α*, and IL-1*β* [33]. In addition, activated microglia play a role in inhibiting inflammatory response and promoting neuronal survival and regeneration by secreting anti-inflammatory factors IL-4, IL-10, and BDNF [34]. Depressed rats were treated with the drug to decrease the levels of TNF-*α* and IL-6 and increase the levels of IL-4, IL-10, and BDNF in the brain. The symptoms of depressed rats also improved [35]. BDNF is a member of the neurotrophic factor family, which plays an important role in nerve growth, differentiation, and repair. The expression of BDNF in the cortex of patients with PSD is negatively correlated with IL-6, TNF-*α*, and IL-1*β* and positively correlated with IL-10 [36]. The results of the present study showed that Flu could inhibit the phosphorylation of NF-*κ*B and I*κ*B-*α* proteins in the hippocampus, thereby reducing the levels of IL-6, TNF-*α*, and IL-1*β* inflammatory factors and restoring those of IL-4, IL-10, and BDNF. Compared with Flu, XNJY could regulate the NF-*κ*B and I*κ*B-*α* signal axis of the cortex and hippocampus, reduce neuroinflammatory response, and protect brain neurons.

Inflammation caused by stroke has been shown to affect synaptic plasticity [37]. The change in synaptic plasticity is an important pathological factor in the onset of depression and PSD [38]. Accompanied by the activation of inflammation, the levels of pro-inflammatory factors (such as IL-6, TNF-*α*, and IL-1*β*) in the brain and peripheral blood increase, and the elevated IL-1*β* and TNF-*α* levels participate in the regulation of NF-*κ*B and the arachidonic acid cascade [39]. Meanwhile, the activated microglia release nitric oxide, which prevented the reuptake of glutamate at the presynaptic site, resulting in excessive glutamate in the synaptic cleft and the activation of NMDA receptors. Amino acid levels could produce excitotoxicity, resulting in a decrease in synaptic markers and loss of neurons [40]. Studies have shown that autopsy of patients with bipolar disorder and schizophrenia showed upregulation of brain neuroinflammation markers and arachidonic acid cascade markers and decreased synaptic markers [41]. SYN is a calcium-binding acid glycoprotein that specifically exists on the membrane of nerve presynaptic vesicles. It directly participates in synapse formation and indirectly reflects the number of synapses and their transmission efficiency [42]. PSD-95 is a member of the membrane-associated guanylate kinase family. It is located in the dense postsynaptic zone, and it is one of the most abundant proteins in the dense postsynaptic substance. In the process of neuron maturation and synapse formation, PSD-95 combines with glutamate receptors, ion channel receptors, and cytoplasmic proteins through its different domains to form couplings, which participate in the regulation of neuronal synaptic plasticity [43]. In the present study, the protein levels of PSD-95 and SYN in these regions of the PSD group were significantly reduced, and treatment with different doses of XNJY and Flu could restore these indicators in the cortex and hippocampus, indicating that XNJY and Flu may exert antidepressant effects by improving synaptic-associated proteins.

In short, XNJY decoction, a TCM complex, could reduce neuronal damage; improve depression-like behavior in rats; inhibit the activation of NF-*κ*B/I*κ*B-*α* pathway; downregulate IL-6, TNF-*α*, and IL-1*β* inflammatory cytokine levels; restore IL-4, IL-10, and BDNF levels; and improve synaptic plasticity-related proteins including PSD-95 and SYN. The results of this study indicated that reducing inflammation and improving synaptic plasticity may be important mechanisms for XNJY to resist depression. The therapeutic effects of XNJY were found in the cortex and hippocampus. However, a part of the effect of Flu was only observed in the hippocampus. This multisite antidepressant effect reflected the multitarget therapeutic effect of traditional Chinese medicine to a certain extent. Therefore, XNJY decoction is expected to become a candidate drug for the treatment of PSD.

## Figures and Tables

**Figure 1:** XNJY increases the body weight of PSD model rats and improves depression-like symptoms. (a) Timetable of experimental procedures. (b) Weight measurement. (c) Sucrose preference test. (d) Forced swimming test. ((e), (f)) Open-field test. Data are expressed as mean ± standard deviation, and multiple comparison analysis is based on analysis of variance. *P* < 0.05 is considered statistically significant. ^*∗∗*^*P* < 0.01, versus sham group; ^##^*P* < 0.01, versus PSD group.

**Figure 2:** XNJY reduces nerve damage caused by PSD. (a) Damage to cortex and hippocampus neurons. (b) Cortex and hippocampal quantitation of Nissl-stained neurons. Cor: cortex; Hip: hippocampus. Data are expressed as mean ± SEM. Multiple comparison analysis is based on analysis of variance. *P* < 0.05 is considered statistically significant. ^*∗∗*^*P* < 0.01, versus sham group; ^##^*P* < 0.01, versus PSD group.

**Figure 3:** XNJY reduces inflammation in PSD model rats. Measurement of IL-6 (a), TNF-*α* (b), IL-1*β* (c), IL-4 (d), IL-10 (e), and BDNF (f) levels in the rat cortex and hippocampus by ELISA. Cor: cortex; Hip: hippocampus. Data are expressed as mean ± standard deviation. Multiple comparison analysis is based on analysis of variance. *P* < 0.05 is considered statistically significant. ^*∗*^*P* < 0.05 and ^*∗∗*^*P* < 0.01, versus sham group; ^#^*P* < 0.05 and ^##^*P* < 0.01, versus PSD group.

**Figure 4:** XNJY regulates the NF-*κ*B/I*κ*B-*α* pathway in PSD model rats. Western blot levels of p-NF-*κ*B, NF-*κ*B, p-I*κ*B-*α*, and I*κ*B-*α* in the cortex (a) and hippocampus (b). Quantitative protein levels of p-NF-*κ*B/NF-*κ*B and p-I*κ*B-*α*/I*κ*B-*α* in the cortex (c) and hippocampus (d). Cor: cortex; Hip: hippocampus. Data are expressed as mean ± standard deviation. Multiple comparison analysis is based on analysis of variance. *P* < 0.05 is considered statistically significant. ^*∗*^*P* < 0.05 and ^*∗∗*^*P* < 0.01, versus sham group; ^##^*P* < 0.01, versus PSD group.

**Figure 5:** XNJY modulates synapse-related proteins in PSD model rats. Protein expression levels of PSD-95 and SYN in the cortex (a) and hippocampus (b). Quantitative protein levels of PSD-95 and SYN in the cortex (c) and hippocampus (d). Cor: cortex; Hip: hippocampus. Data are expressed as mean ± standard deviation. Multiple comparison analysis is based on analysis of variance. *P* < 0.05 is considered statistically significant. ^*∗∗*^*P* < 0.01, versus sham group; ^#^*P* < 0.05 and ^##^*P* < 0.01, versus PSD group.

## Data Availability

The data used to support the findings of this study are available from the corresponding author upon request.
